# Activation of Nuclear Factor Kappa B (NF-kB) Signaling Pathway Through Exercise-Induced Simulated Dopamine Against Colon Cancer Cell Lines

**DOI:** 10.7759/cureus.46624

**Published:** 2023-10-07

**Authors:** Dhanushree Baranikumar, Meenakshi Sundaram Kishore Kumar, Venkataramanan Natarajan, Lavanya Prathap

**Affiliations:** 1 Department of Anatomy, Saveetha Dental College and Hospitals, Saveetha Institute of Medical and Technical Sciences, Saveetha University, Chennai, IND

**Keywords:** exercise, sustainable development, good health and well-being, inflammatory pathway, dopamine, colon cancer prevention

## Abstract

Introduction

Dopamine is an important neuroregulatory hormone and is secreted during exercise. Its role in physiological regulation is not fully uncovered. Recent studies showed that it suppresses inflammation. Colon cancer is one of the most predominant cancers in the population and is influenced by prolonged inflammation. The anti-inflammatory effect of dopamine using the colon cancer model was analyzed in KB cells.

Methods

KB cells were cultured using Dulbecco's Modified Eagle Medium* *and Inhibitory Concentration- 50 (IC_50_) was determined by 3-[4,5-dimethylthiazol-2-yl]-2,5 diphenyl tetrazolium bromide assay. BCl-2, tumour necrosis factor-α (TNF-α), nuclear factor kappa- B (​​​​​NF-kB), and interleukin (IL)-6 were assessed using reverse transcription polymerase chain reaction (RT-PCR)(at 50 and 100 µg/ ml < IC_50_). Schrödinger was used for docking analysis using nuclear factor Kappa B (NF-kB) (Protein Data Bank: 5T8O) and dopamine (CID 681).

Results

Results were represented as mean ± standard deviation and statistically evaluated. Dopamine showed severe growth inhibition in KB cells (IC_50_- 225±3.1µg/ ml). It downregulated the expression of BCl-2, NF-k, and IL-6, but increased TNF-α expression. Dopamine bonded with NF-kB by two hydrogen bonds with aspartic acid​​-53and alanine-54, respectively).

Conclusion

The present study revealed that dopamine has a significant anti-cancer potential by blocking NF*-*kB* *pathways in KB cells.

## Introduction

Exercise has been proven to be highly connected with inhibiting the occurrence of different chronic diseases, particularly a variety of human cancers. Many clinical trials accompanied by meta-analyses revealed that exercise greatly reduces colorectal cancer (CRC) [1,2]. CRC is the most common cancer type among innumerable populations. Its prognosis increases daily, and it is anticipated to affect* *2.5 million people by 2035 [3]. Colon cancer, particularly, is at high risk in the population because it is characteristically enhanced by several lifestyle modifications [4]. Several populations changed their traditional food habits and mainly depend on fat-rich foods nowadays [5,6]. A high proportion of red meat, beverages, sugar-rich diets, and fewer vegetables in food preparations increases the chances of colon cancer. In addition, smoking, consumption of hot drinks, and a sedentary lifestyle directly prolong inflammation and result in chronic diseases [7,8]. Those metabolic changes lead to metabolic dysfunction, inflammation, and oxidative stress. Due to the complexity of mechanistic signaling in these physiological networks, colon cancer remains a hard challenge for therapeutic discovery [9]. Chemotherapy, surgery, and radiotherapy are three ways to treat colon cancer, but, many associated factors such as side effects, and tumor recurrence usually limit such therapeutic goals [10]. Since in most cases the diagnosis is done at the level of metastasis, the treatments seem to be ineffective for these patients in prolonging their survival [11,12].

On another side, physical training and exercise have been shown to prevent or inhibit malignancies in different types of cancers, including proximal and distal colon, endometrial, prostate, breast, lung, gastroesophageal, renal, and pancreatic cancer [3]. Exercise and the associated secreting molecules disturb the growth of malignancies by reducing inflammation and inhibiting the cancer-signaling pathways [1, 5]. Several studies showed that exercise decreases the mitogenic signals based on different animal models. Exercise increased the expression of p53 and inhibited the tumor-suppressing genes. Exercise also reduced the levels of hyper-phosphorylated retinoblastoma protein in a mouse model of breast cancer [13]. Dopamine (DA), a type of neurotransmitter and regulator by central and peripheral brain cells, is released as a result of exercise. As a crucial signaling molecule for motor neurons, memory processing, and other related cognitive tasks, it also aids in the chemical homeostasis of the nervous system.Recent research has indicated that dopamine plays a significant role in inhibiting the development of cancer [14]. Additionally, malignant cells have a certain amount of dopamine and their growth is slowed down when the concentration of dopamine rises. It also reduced chronic stress-associated angiogenesis and decreased tumor growth [15].

Mitochondria have their own DNA that varies significantly from genomic DNA and regulate the cell's energy currency (adenosine triphosphate (ATP))*.* They have the ability to organize reactive oxygen species (ROS) and their associated inflammatory, apoptotic, and anti-apoptotic pathways. The chemotherapeutic drugs that target mitochondria regulate their membrane potential (mitochondrial transmembrane potential (MTP)) and modify Bax/BCl-2 expression. NF-kB (Nuclear-Factor-kappa-B) increases inflammation and its overexpression leads to cancer growth by decreasing the Bax/BCl-2 ratio [16]. NF-kB positively contributes to cancer growth by expressing IL6, and TNF-α. Dopamine inhibits NF-kB in different cancer types, including breast, prostate, and lung cancer cells [17]. The possibility of dopamine as an alternative medication for the treatment of colon cancer and its anti-inflammatory nature was analyzed in this study.

## Materials and methods

Cell viability assay - MTT assay

The MTT (3-[4,5-dimethylthiazol-2-yl]-2,5 diphenyl tetrazolium bromide) method was used for assessing the KB cell (procured from the National Centre for Cell Sciences, Pune, India) viability under dopamine treatment. KB cells are keratin-forming tumor cells, a sub-cell line of HeLa cells. Briefly, 10^3^/well were cultured (with Dulbecco's Modified Eagle Medium** **(DMEM) (10% Fetal Bovine Serum (FBS), 1% penicillin and streptomycin)) and incubated for 24 h, 37°C, 5% CO_2_) to enhance the cell adherence. 80% confluency was ensured for the commencement of the experiment (0, 50, 100, 250, and 500 µg/ml, dopamine) in dimethylsulfoxide (DMSO) (0.1% as maximum). Cell viability was checked after 48 h, compared with the untreated cells. IC_50_ was calculated using the probit method [18,19]. A protein denaturation (in vitro) assay was done by adopting the previous method** **(Varshan et al., (2022)** **[20]).

RT-PCR reaction

After being exposed to dopamine for 48 hours, KB cells were treated with the TRIzol reagent to isolate the total RNA from them (Takara Bio, Dalian, China). Using a Prime Script RT Reagent Kit (Takara, New Delhi, India), for synthesizing, complementary deoxyribonucleic acid (cDNA) was reverse-transcribed. For the amplification, an Mx3005P Real-Time Polymerase Chain Reaction System was employed (Agilent, Santa Clara, USA), and the kit's directions were followed for the quantitative polymerase chain reaction (Q-PCR)** **experiment. The messenger ribonucleic acid (mRNA) expression levels of each gene were normalized to the RNA of glyceraldehyde 3-phosphate dehydrogenase ​​​​​(GAPDH)using the cycle threshold (2CT) method. The primers were produced by Shanghai, China-based Invitrogen [21].

Molecular docking analysis

The structure of dopamine (PubChem database with CID 681) and NF-kB (Protein Data Base (PDB:5T8O) were retrieved. The Schrödinger software suite (Schrödinger Maestro 11.2 version, New York, USA) was used to prepare the Epik (rapid and robust pKa predictions) states and to optimize the ligand. The docking was carried out using the extra precision method (XP) and the Glide score (docking score given by Glide software, a subset of Schrödinger) was calculated and expressed as kcal/mol [22].

Statistical analysis

The significant value was confirmed using one-way (Newman-Keuls post hoc test) and two-way ANOVA (Bonferroni post hoc test).

## Results

One of the primary factors in the development of cancer is persistent inflammation. Its involvement in the development and spread of colon malignancies has been thoroughly investigated. Dopamine inhibited inflammatory effects on KB cells. On KB cells, dopamine decreased the expression of inflammatory genes such as TNF-α, NF-B, and p38 but enhanced the expression of Bax.

Effect of dopamine on cell viability

Using the MTT assay, the cytotoxic effect of dopamine was investigated. For the investigation, various concentrations, such as 0, 50, 100, 250, and 500 µg/ml were employed. In comparison to controls, the findings demonstrated that dopamine exhibited dose-dependent cytotoxicity with KB cells (Figure 1). The IC_50_ values of doxorubicin and dopamine were calculated as 125.41±1.56 and 225±3.1 µg/ml, respectively. The expression of pro and anti-inflammatory genes was analyzed in two concentrations, 50 and 100 µg/ml, respectively.

**Figure 1:** Effect of doxorubicin and dopamine on KB cells. Different concentrations (50-500 µg/ml) of respective drugs treated with KB cells for MTT assay. The x-axis represents the log concentration (µg/ml) and the y-axis represents cytotoxicity (%) Two-way ANOVA was carried out with Bonferroni post hoc test. (* representing statistical significance, * represents p<0.05, ** represents p<0.005, *** represents p<0.001) Image Credit: Lavanya Prathap

Dopamine inhibited BCl-2 mRNA expression on KB cells

The mRNA expression of the BCI-2 gene on dopamine-treated KB cells was assessed using qPCR. Two concentrations, 50 and 100 µg/ml, were used based on IC_50_ for the study. At 100 µg/ml, dopamine leads to decreased BCl-2 expression in KB cells. The BCl-2 decrease was more at 100 µg/ml than at 50 µg/ml. Thus, decreased BCl-2 expression was dose-dependent concerning dopamine treatment. As a result, the increased gene expression was dose-dependent (Figure 2).

**Figure 2:** Dopamine inhibited the expression of BCl-2 mRNA on KB. Drug concentration (log) is shown on the x-axis, while fold change over control is shown on the x-axis, and yellow represents control. Bax expression in higher concentration 100 µg/ml. One-way ANOVA – Newmann-Keuls post hoc test (* represents statistical significance, ** represents p<0.005, ns=not significant). Image Credit: Lavanya Prathap

Dopamine decreased TNF-α mRNA expression in KB cancer cells

In a dose-dependent manner, the dopamine decreased mRNA expression of TNF-α in KB cells. The study utilized two concentrations, 50 and 100 µg/ml. The cancer cells showed more decreased levels of TNF-α at a concentration of 100 µg/ml than they did when treated with 50 µg/ml. The findings demonstrated that, in comparison to control, there was a significant decrease (about a four-fold decrease) in the mRNA expression of TNF-α. Additionally, at a dose of 50​ µg/ml**​​​​​​**, NF-kB mRNA expression decreased significantly in comparison to control. The gene expression modification was consequently dose-dependent in treated cells compared with the control (Figure 3).

**Figure 3:** Dopamine reduced the expression of TNF-α mRNA on KB cells The fold change over control is displayed on the y-axis, while drug concentration (log) is displayed on the x-axis. TNF-α expression was found with a statistically significant reduction at a concentration of 100 µg/ml compared to the control. * represents statistical significance, * represents p<0.05, ** represents p<0.005, *** represents p<0.001. TNF-α, tumour necrosis factor alpha Image Credit: Lavanya Prathap

Dopamine inhibited NF-kB mRNA expression on the KB cells

The ratio of the NF-kB in KB cells treated with dopamine was analyzed using qPCR. The expression was in a dose-dependent manner. At 50 µg/ml, dopamine showed a significantly reduced NF-kB expression compared to the control (Figure 4).

**Figure 4:** Effect of dopamine on the expression of NF-kB mRNA on KB cells. On the y-axis is the fold change compared to the control, and on the x-axis is the drug concentration (log). * represents statistical significance, * represents p<0.05, ** represents p<0.005, *** represents p<0.001 Image credit: Lavanya Prathap

Our results indicated that dopamine decreased the inflammation by attenuating the pro-inflammatory markers such as NF-kB and BCl-2. Meanwhile, it increased the expression of TGF-α (T cell growth factor - α) in a dose-dependent manner.

Molecular docking

The protein structure (PDB: 5T8O), which contains the structure of murine NF-kB and kinase-bound imidazolbenzoxepin molecule, was downloaded from the PDB databank (Figure 5). After the protein structure was refined by the protein wizard, the binding site detector was utilized to identify the protein's binding pockets. The confirmation and orientation of the ligand-inhibitor complex at the active or docking site is an important concept for drug discovery. In the present study, the Schrödinger docking software was used; the results are presented in Figure 5 and Figure 6. Figure 5 presents the protein structure. The NF-kB-dopamine complex's expected binding-free energy was discovered to be -2.456 kcal/mol (Figure 6). The pose with the highest docking energy is represented in Figure 6. Dopamine bonded with NF-kB with two intramolecular hydron bonding (Figure 6a). Using the LigPlot+ program and the BIOVIA DS Visualizer (both of them a subset software of the Schrödinger suite), we also investigated the presence of intermolecular interactions in protein-ligand complexes in this study (Figure 6b-6c). Dopamine made two hydrogen bonds with NF-kB through two amino acids, aspartic acid (ASP-55) and alanine (ALA-54).

**Figure 5:** Structure of NF-κB (PDB - 5T80). Structure of NF-κB docked with dopamine for analyzing its protein-ligand binding properties. Image credit: PDB ID: 5T80, Lavanya Prathap.

**Figure 6:** Molecular binding of dopamine with NF-κB. (a) Structural conformity of protein-ligand binding.  (b) The binding of dopamine led to electrostatic cloud formation. (c) Ligand view inside the protein.  (d) Formation of hydrogen bond Image credit: Lavanya Prathap

## Discussion

The dopamine pathway has lately come to light as a possible target in anticancer medicines, drawing on decades' worth of evidence linking the dopamine effect and cancer. Repurposing dopaminergic medications has considerable benefits for patients [23]. Exercise is one of the easiest ways to gain dopamine at the tissue level. Despite this, a thorough investigation into the potential uses of this therapy approach in cancer is warranted given the abundance of evidence connecting DA to cancer and non-tumor cells in the tumor microenvironment. Summarizing the prior empirical research on the reciprocal relationship between dopamine, we found strong evidence for strong anti-cancer activity of dopamine through the regulation of NF-κB in KB, colon cancer cells [24]. Dopamine decreased pro-inflammatory markers more than the control.

The relationship between an increase in extracellular dopamine and NF-κB activation and inflammation reveals certain intracellular targets that may be exploited to discover novel targets in colon cancer cells for effective treatment strategies. Our results are concordant with the previous studies [25-27]. DA was shown to reduce tumor growth, metastasis, and tumor angiogenesis [25]. Similar to the present study, Wu et al. (2020) showed that DA blocked the expression of NF-κB and reduced inflammation [27]. Prolonged inflammation stimulates the immune cells to secret a lot of inflammatory cytokines (such as IL-1, IL-6, and TNF-α) [28]. Our results showed that DA could suppress a few of those pro-inflammatory markers in KB cells. Previously, we showed that dopamine substantiated BCl-2 in A549 cells[4].

Dopamine has shown a strong inhibition of inflammation on cancer sites. Different biochemical mechanisms had been reported previously. Such inhibition of inflammatory pathways seemed to enhance its therapeutic efficacy on pancreatic cancer. It deprived the cyclic adenosine monophosphate (cAMP) and inhibited the protein kinase A/protein 38 (PKA/p38) signaling by activating the dopamine D2-like receptor-4 (DRD4) receptor. DRD4 is one of the dopamine family receptors (DRD1-DRD5). Thus, it inhibited the activation of tumor-associated macrophages also [29]. Dopamine inhibits NF-κB by activating DRD2, DRD3, DRD4, and DRD5 receptors. DRD2 activation led to gastric cancer reduction in previous studies [30]. In contrast, Kline et al. (2018) showed that knockout of DRD2 in colon cancer did not alter properties and had an independent mechanism [30].

## Conclusions

Our findings further imply that dopamine might be an endogenous bioactive substance with anti-inflammatory qualities, making it a potential treatment for malignant colon cancer and other pathological disorders caused by inflammation through NF-κB signal.
